# A Magnetically Capsule Robot for Biomedical Application

**DOI:** 10.1155/2022/2233417

**Published:** 2022-07-21

**Authors:** Qiang Fu, Xi Zhang, Songyuan Zhang, Chunliu Fan, Zhuocong Cai, Lili Wang

**Affiliations:** ^1^Tianjin Key Laboratory for Control Theory & Application in Complicated Systems, Tianjin, China; ^2^School of Electrical Engineering and Automation, Tianjin University of Technology, Tianjin, China; ^3^State Key Laboratory of Robotics and System, Harbin Institute of Technology, Harbin, China; ^4^Tianjin Hospital of ITCWM Nankai Hospital, Tianjin, China

## Abstract

Magnetic-driven capsule robot has been widely studied due to its advantages of safety and reliability. However, when doctors carry out clinical examination, the capsule robot cannot achieve the ideal control effect due to the influence of the external magnetic field air gap. This paper is based on the kinetic energy theorem, combined with the principle of spiral mechanism in mechanical design foundation to construct a calculation method of energy utilization and to improve the control effect of capsule robot, suitable for the human gastrointestinal tract precise control of capsule robot to perform a variety of complex tasks. By calculating the energy utilization rate of the capsule robot under the control of external magnetic field, the method can improve the energy utilization rate by improving the equation parameters, so that the capsule robot can run according to the doctor's ideal performance in practical application. Based on the analysis of the magnetic driven screw capsule robot, the model of the utilization rate of the external magnetic field of the capsule robot is established, and the fluid simulation of the capsule robot is carried out by using the method of computational fluid dynamics. The simulation results and experimental results show that the control effect of capsule robot can be improved by calculating the energy utilization rate of the robot, which is of great significance to human clinical examination and treatment.

## 1. Introduction

Gastroscopy is an essential method for the diagnosis of internal gastrointestinal diseases. The traditional gastrointestinal endoscopy needs a manual operation, which can easily cause gastrointestinal tissue damage. It may even lead to infection or gastrointestinal bleeding, causing many people to give up the diagnosis and treatment of the gastrointestinal tract by traditional endoscopy [1–3]. The cure rate of gastrointestinal diseases is closely related to the time of discovery: the earlier the discovery, the more conducive to the treatment and recovery of the disease. Capsule robot has been widely studied because of their advantages, such as being safer, comfortable, and painless [4–6]. Compared with a traditional plug-in electronic endoscope, a capsule robot avoids the hidden dangers such as cross-infection and secondary trauma of traditional tubular endoscopes, reduces the pain in the inspection process, and widens the inspection field and detection breadth [7–9].

Capsule robot detection technology has developed rapidly; Israeli medical technologies pioneered the “M2A” capsule robot for gastrointestinal examinations [10–12]. Chongqing Jinshan Technology and Japan's Olympus have launched their capsule robots “OMOM” [13] and “Endo Capsule” [14]. However, these capsule robots can only rely on intestinal peristalsis to change the position in the body [15–17], and this passive motion mode cannot accurately detect the lesions, which is prone to missed diagnosis and misdiagnosis. Therefore, the capsule robot that can realize active movement has become the inevitable development trend of intestinal detection.

Fu et al. studied an external field-driven cable-free microrobot with bionic swimming characteristics. By changing the driving frequency of the time-varying oscillating magnetic field, the film tail fin is driven to fluctuate to achieve more flexible movement in the intestines and stomach full of body fluids [18]. Fu et al. proposed a soft capsule robot for the continuous and stable control of the capsule robot in the body. Under the control of the external magnetic field, the motion is carried out in the rolling motion mode so that the motion is stable, continuous, and controlled in the gastrointestinal tract [19]. Fu et al. proposed a magnetically driven microrobot with a covered propeller structure, which improved the efficient propulsion performance of the capsule robot and reduced the harm to the stomach [20]. In addition, a new kind of rotating magnetic field hybrid microrobot is proposed, which combines the spiral structure with the biomimetic fin tail, so that the two motions can be controlled independently without interference, and the flexible motion with multiple degrees of freedom is realized [21]. However, the above literature does not consider whether the capsule robot can always maintain accurate and efficient control in a complex environment full of fluid.

To solve the above problems, this paper proposes a calculation method to improve the control of magnetic-driven spiral capsule robot, which is used in the visualization research of capsule robot control and improves the control effect of capsule robot. According to the kinetic energy theorem and the principle of spiral mechanism in mechanical design, the energy utilization equation is constructed to calculate the actual energy utilization percentage of the capsule robot. The results are used to reflect and analyse the motion control effect of capsule robot. This method can verify the control effect of capsule robot in actual medical process and adapt to complex gastrointestinal environment.

The structure of this paper is as follows: Firstly, the structure of the magnetically driven capsule robot is introduced. Then, the dynamic model of the robot is established, and the method of improving the robot's motion performance is analysed. Then, the feasibility of the method is verified by simulation and experiment. Finally, this paper summarizes and looks into the future.

## 2. System Configuration

Integrated console, display, three-axis Helmholtz coil, and 6∗6 magnetic sensor array constitute the remote-control system of the capsule robot (Figure 1(a)) [22]. The three-axis Helmholtz coil and sensor array actuate and locate the capsule robot. The integrated console and display are used for real-time image feedback of the capsule robot working in the human body.

### 2.1. Working Principle

When the patient swallowed the single module or multiple module capsule robot, the capsule robot arrived at the starting position through gastrointestinal peristalsis. At this point, the doctor can observe real-time images in the gastrointestinal tract on display and control the three-axis Helmholtz coil through the integrated console to generate an external rotating magnetic field to drive a single or multiple capsule robot forward or backwards in the patient [23–25]. The integrated console controls the three-axis Helmholtz coil to generate an external rotating magnetic field, driving the capsule robot forward or backwards.

Furthermore, use a 6∗6 magnetic sensor array as the positioning system, real-time positioning of the position and orientation of the capsule robot, to achieve accurate control of the capsule in the complex gastrointestinal environment, complete inspection, treatment, and other tasks.

### 2.2. Robot Structure

The capsule robot consists of modules with a polyethene shell and an O-ring magnet. When swallowing a multimodule capsule robot, based on the previous research on the motion characteristics of a multimodule capsule robot, the difference of starting and cut-off frequency of each module can be used to realize its separation or whole movement [26–28]. The parameters of capsule robots A, B, and C are used in this paper (Table 1). The overall structure of capsule robot A is shown in (Figure 1(b)), and its internal structure is shown in (Figure 1(c)). If the capsule robot rotates in the patient's body, it must obtain an axial positive magnetic moment generated by the three-axis Helmholtz coil. When the o-type permanent magnet inside the capsule robot rotates, the magnetic moment generated overcomes the resistance moment, resulting in a positive magnetic moment to start the robot. The motion state of capsule robot can be expressed by driving torque *T* in the following equation:

(1) $$\begin{array}{c} T=T_{M}-T_{F}, \end{array}$$

where *T*_*M*_ is the magnetic moment generated by the capsule robot and *T*_*F*_ is the resistance moment generated.

When *T* > 0, it indicates that the capsule robot is in the state of start-up or acceleration. When *T* = 0, it means the capsule robot is in a static or uniform state. When *T* < 0, it indicates that the capsule robot is in the deceleration or stop state [29].

## 3. Dynamic Model

### 3.1. The Analysis of the Force

The dynamics model of the capsule robot is established in the intestinal tract (Figure 2). Cartesian coordinate axes are established, and u_c_ is defined as circumferential velocity and v_a_ as axial velocity. A_1_ and A_2_ are, respectively, the thread spacing and thread width of the capsule robot, and r_1_ and r_2_ are the surface rotation radius of the capsule robot. L is the length of the capsule robot, and p is the pitch of the capsule robot [30]. The force analysis of the capsule robot is as follows:

The motion state of the capsule robot is by the following equation:

(2) $$\begin{array}{c} ma=F_{P}-F_{D}\pm G\mp \rho {gV}_{D}, \end{array}$$

where *F*_*P*_ is propulsion force, *F*_*D*_ is resistance force, *G* is gravity acting on the microrobot, *g* is the acceleration of gravity, and *V*_*D*_ is drainage volume.

The resistance force *F*_*D*_ equation is expressed as follows:

(3) $$\begin{array}{c} F_{D}=C_{D}\frac{1}{2}\;\rho v^{2}S+\mu_{f}N, \end{array}$$

where *C*_*D*_ is the drag coefficient, *v* is the velocity of the capsule robot, *S* is the cross-sectional area of the simulated pipe, *μ*_*f*_ is the kinematic viscosity coefficient, and *N* is the normal force.

When the capsule robot rotates, the projection of circumferential velocity *u*_*c*_ and axial velocity *v*_*a*_ in *X* and *Y* directions is defined by the following equations:

(4) $$\begin{array}{c} W=u_{\text{c}}\sin\theta -v_{a}\cos\theta , \end{array}$$

(5) $$\begin{array}{c} V=u_{\text{c}}\cos\theta +v_{a}\sin\theta , \end{array}$$

where *W* and *V* represent the velocity component of the projection capsule robot relative to the fluid in *X* and *Y* directions, respectively, and *θ* represents the helix angle.

In order to facilitate calculation, based on previous research results on capsule robot kinematics [18–22], Equations (6) and (7) of axial propulsion force and resistance are derived from Equations (4) and (5):

(6) $$\begin{array}{c} F_{\text{pro}}=F_{y}\sin\theta -F_{x}\cos\theta , \end{array}$$

(7) $$\begin{array}{c} F_{\text{res}}=F_{y}\cos\theta +F_{x}\sin\theta , \end{array}$$

where *F*_pro_ represents the axial propulsion force in motion and *F*_res_ represents the axial resistance in motion.

In dynamic analysis, axial thrust *F*_pro_ decreases with increasing velocity. When the axial propulsion force is equal to the axial resistance, the acceleration of the capsule robot is 0, and the speed is the maximum, and it moves stably at this speed.

### 3.2. Energy Conversion Formula

According to the law of energy conservation, the motion performance of the capsule robot in various complex environments is considered. When the capsule robot moves from point *A* to point *B*, the total energy *W* is equal to the change of kinetic energy ∆K, where point *A* and point *B* are two uniform points, as follows:

(8) $$\begin{array}{c} W=\int_{A}^{B}\text{d}W=\int_{B}^{A}\bar{F}\cdot d\bar{r}=\Delta K. \end{array}$$

According to the energy conservation law, the equation of kinetic energy under ideal ∆Ki and actual ∆Kr conditions is defined by Equations (9) and (10). It follows that a change in velocity affects kinetic energy. Not all energy is converted into kinetic energy in the actual process, and part of the energy will be converted into heat energy due to resistance [31]:

(9) $$\begin{array}{c} \Delta K_{i}=\frac{1}{2}{mv}_{iB}^{2}-\frac{1}{2}{mv}_{iA}^{2}, \end{array}$$

(10) $$\begin{array}{c} \Delta K_{r}=\frac{1}{2}{mv}_{rB}^{2}-\frac{1}{2}{mv}_{rA}^{2}. \end{array}$$

The percentage of actual energy utilized *η* by the capsule robot in the process of movement is shown in the following equation:

(11) $$\begin{array}{c} \eta =\frac{\Delta K_{r}}{\Delta K_{i}}\times 100\%, \end{array}$$

The shell of capsule robot adopts screw structure (Figure 3(a)). So, the principle of screw mechanism in mechanical design foundation can be used to analyse the capsule robot [32]. Part of the screw structure (Figure 3(b)) and the force analysis is carried out on the inclined plane of the screw thread (Figures 3(c) and 3(d)). The work required by the capsule robot to move forward *W*_*r*_ is shown in the following equation:

(12) $$\begin{array}{c} W_{r}=G*S_{\text{r}}=G*2\pi {\text{r}}_{1}*\tan\theta , \end{array}$$

where *S*_*r*_ is the actual horizontal movement distance of the capsule robot.

The work done to make the capsule robot move forward *W*_*i*_ is shown in the following equation:

(13) $$\begin{array}{c} W_{i}=G*S_{\text{i}}=G*2\pi r_{1}*\tan\left(\varphi_{s}+\theta \right), \end{array}$$

where *S*_*i*_ is the ideal horizontal movement distance of the capsule robot and *φ*_*s*_ is the dynamic friction angle.

Therefore, the energy utilization rate *η* of the capsule robot can be deduced to the following equation:

(14) $$\begin{array}{c} \eta =\frac{W_{\text{r}}}{W_{i}}=\frac{S_{\text{r}}}{S_{i}}=\frac{\tan\theta }{\tan\left(\varphi_{s}+\theta \right)}. \end{array}$$

According to Equation (14), the percentage of energy utilized by the capsule robot during the actual movement is equal to the percentage of the actual and ideal moving distance. The actual distance is the horizontal moving distance of the capsule robot, and the ideal moving distance is a multiple of the pitch, as shown in the following equation:

(15) $$\begin{array}{c} \eta =\frac{S_{\text{r}}}{S_{i}}=\frac{vt}{fpt}=\frac{v}{fp}, \end{array}$$

where *v* is the speed of the capsule robot, *f* is the frequency, and *p* is the pitch of the capsule robot.

## 4. Dynamic Analysis

When the capsule robot moves in a fluid-filled pipe, because many variables are affecting the motion, in order to accurately simulate the motion of the capsule robot in the optimal state, a single variable control method is used to simulate the fluid of the capsule robot. The capsule robot model has dynamically meshed. Since the human intestine is similar to a cylinder, we built a cylinder with the same length as the actual experiment as the intestine in the simulation, about 500 mm. The inlet and outlet of the intestine and the direction of forwarding flow velocity are set. In the fluid simulation, the horizontal movement of the capsule robot is studied. In order to reduce the influence of other factors, vertical forces such as gravity and buoyancy are ignored.

In the fluid simulation, a dynamic model with a rotating speed range of 0-150 rad/s and geometric parameters of 10 rad/s is established to carry out the whole fluid simulation at standard atmospheric pressure. Fluid simulation is carried out for capsule robots A, B, and C in Table 1, respectively, and the motion states of these three capsule robots in the pipeline are analysed from dynamics. Due to the different pitches of the three capsule robots, their cross-section shapes are different. Considering that the position of the capsule robot is unchanged in the simulation process, the influence of resistance can be ignored.

Set capsule robots A, B, and C at the same speed, observe their water inlet surface, and get the speed simulation diagram (Figure 4). When the three capsule robots rotate at the same speed, the shorter the pitch, the faster the fluid around the capsule robot. Observe the velocity simulation of capsule robots A, B, and C in the middle plane (Figure 5). It can be seen that at the same speed, the velocity of the three capsule robots is greater than the inlet surface, and the shorter the pitch, the greater the fluid velocity of the middle part of the capsule robot. By observing their outlet surfaces at the same speed, the velocity simulation diagram (Figure 6), it can be seen that the color distribution of the capsule robot at the outlet surface of the capsule robot is not uniform, indicating that the fluid growth rate of different parts of the capsule robot is not uniform at the same speed. By comparing the fluid cloud images of three different parts of the capsule robot, it can be seen that different parts of the capsule robot are affected by different fluid velocities and have different influences on its surroundings. This also lays a foundation for subsequent experiments, especially for selecting capsule robots, which can select the corresponding pitch according to different medical tasks [33].

## 5. Experimental Results

The experimental platform was used to test the performance of capsule robot (Figure 7). The motion direction and rotation speed of the capsule robot in the liquid-filled pipe are controlled by adjusting the frequency and direction of the magnetic field. When the upper computer outputs the drive signal, the three-axis Helmholtz coil generates a uniform rotating magnetic field, and the capsule robot placed in the middle of the magnetic field gets the energy to drive the rotation.

### 5.1. Robot Kinematic Characteristic Experiment

By observing the capsule robots, A, B, and C (Figure 8), it can be seen that the three differences only lie in the pitch, which is 10 mm, 7 mm, and 5 mm, respectively. The capsule robots are put into the acrylic tube filled with water, respectively, to conduct the characteristic motion experiment, and the start-up and cut-off frequencies of capsule robots A, B, and C under different currents are measured (Figures 9 and 10). The experimental results show that the start-up and cut-off frequencies of the capsule robot vary with the current. In the same current, the shorter the pitch of the capsule robot, the lower the start-up frequency, the higher the cut-off frequency. The difference between start-up and cut-off frequency simultaneously controls of multiple capsule robots or separate control in the same environment. This is to achieve the movement control of the multimodular capsule robot in the intestinal tract to better complete the task of medical treatment.

Adjust the input current to 0.5 A, and the velocities of capsule robots A, B, and C are measured at different frequencies. The external control signal adjusts the frequency from 0 Hz to 25 Hz (Figure 11). The experimental results show that the velocity increases with the increase of frequency. At the same frequency, the larger the pitch of the capsule robot, the faster the speed, the more energy is converted into kinetic energy, and the less energy is consumed to overcome resistance.

### 5.2. Energy Utilization Percentage Experiment of Capsule Robot

The established capsule robot model is placed in the simulation environment for experiments. Parameters are set at standard atmospheric pressure to simulate the movement of the capsule robot, and the velocity of movement at different frequencies is collected and put into Equation (15) to calculate the energy utilization rate of the capsule robot in the simulation environment. Compared with the energy utilization rate obtained in the actual motion characteristic experiment, the energy utilization rate curve of the capsule robot in the process of motion is obtained (Figure 12). The two curves of the simulation experiment and the actual experiment fluctuate around the starting frequency, but the overall trend is consistent. With the increase of frequency, the energy utilization rate increases, indicating that the control effect of the capsule robot is better. Then, the velocity of capsule robots B and C collected in the motion characteristic experiment is substituted into the following.

Equation (15) was used to obtain the energy utilization curve of capsule robots A, B, and C (Figure 13). When the frequency is constant, the smaller the capsule robot pitch is, the higher the energy utilization ratio is, which verifies the feasibility of the energy utilization ratio equation.

The energy efficiency equation reflects the accuracy of the motion control effect of the capsule robot and is also related to the flexibility of the motion control of the capsule robot. When the capsule robot controls the flexibility, the measured velocity is more accurate and the calculated energy utilization rate is more accurate. Therefore, round-trip movement experiment and multidimensional space movement experiment should be carried out to verify that the capsule robot can be flexibly controlled in human body.

In the round-trip movement experiment (Figure 14), the control magnetic field is rotated clockwise in the *Y*‐*Z* plane until it stopped at 280 mm for 4 s. The counter clockwise rotation of the magnetic field returns the capsule robot 110 mm. The experimental results show that the capsule robot can start and stop flexibly according to different medical tasks. In the multidimensional space movement (Figure 15), the feasibility of the capsule robot moving in multidimensional space needs to be verified by horizontal movement, vertical movement, and 70° horizontal *Y*-axis movement, respectively, due to the complex actual intestinal environment of human body. The results show that the capsule robot can obtain the propulsion force by adjusting the rotating magnetic field, which verifies that the capsule robot can be flexibly controlled in multiple directions of the three-axis Helmholtz coil.

## 6. Conclusion

This paper presents a method to improve the control effect of magnetic driven spiral capsule robot. The capsule robot that tested the method is made of a shell made of polyethylene plastic and an O-ring magnet. By measuring the start-up and cut-off frequency of the capsule robot, determine the frequency control range of single or whole movement of the capsule robot. By comparing the simulation and actual experiment of capsule robot with the same pitch and the actual experiment of capsule robot with three different pitches, the curves obtained all show an upward trend, which verifies the different energy utilization results with different parameters in the equation, indicating the feasibility of this method. According to the experimental results, the energy efficiency of the capsule robot will be improved with the change of the size of the capsule robot's pitch. However, the increase of the pitch of the capsule robot will affect the stability of the motion, so in the future precise control of the capsule robot, the energy utilization equation can be considered to improve the control of the capsule robot, while considering the stability of the motion, in order to achieve the ideal control effect.

## Figures and Tables

**Figure 1:** (a) Remote control of the system. (b) Overall structure of capsule robot. (c) Internal structure of capsule robot.

**Figure 2:** Capsule robot model.

**Figure 3:** (a) Overall thread structure diagram. (b) Partial thread structure stress analysis. (c, d) Thread section stress analysis diagram.

**Figure 4:** Simulation of inlet plane velocity profile of different capsule robots at the same rotational speed.

**Figure 5:** Simulation of intermediate plane velocity profile of capsule robot at the same rotational speed.

**Figure 6:** Simulation of exit plane velocity profile of different capsule robots at the same speed.

**Figure 7:** The electromagnetic actuation system.

**Figure 8:** Capsule robots with different pitch.

**Figure 9:** Start-up frequency at different current currents.

**Figure 10:** Cut-off frequency of different currents.

**Figure 11:** Relationship between frequency and velocity of capsule robot at different pitch.

**Figure 12:** Efficiency of capsule robot at different frequencies.

**Figure 13:** The actual working efficiency of three capsule robots at different frequencies.

**Figure 14:** Multiple reciprocating motion.

**Figure 15:** Hyperspatial motion. (a–c) The forward horizontal movement of the *X*-axis; (d, e) the reverse horizontal movement of the *X*-axis; (g, h) locomotion direction is 70° *Y*-axis; (i–k) the vertical movement of the *Z*-axis.

**Table 1:** Capsule robot main parameters.

Symbol	Robot A	Robot B	Robot C
Length of capsule robot (mm)	20	20	20
Radius of capsule robot (mm)	5.5	5.5	5.5
Thread pitch (mm)	10	7	5
Thread height (mm)	2	2	2
Thread width (mm)	2	2	2
Material of body	Polythene	Polythene	Polythene
Weight of magnet (g)	5	5	5
Material of magnet (g)	1.5	1.5	1.5
Magnetization direction	Radial	Radial	Radial
Magnetization direction	NdFeB35	NdFeB35	NdFeB35

## Data Availability

The data used to support the findings of this study are included within the article.
